The article "Evaluation of Tresiba Combined with Six Ingredient Rehmannia Pill in the Treatment of Type 2 Diabetes" was retracted in 2023. Reasons: signs of a paper mill; suspected computer-generated content; unreliable results or conclusions; lack of ethics approval or compliance.

# Evaluation of Tresiba Combined with Six Ingredient Rehmannia Pill in the Treatment of Type 2 Diabetes

**DOI:** 10.1155/2022/2177176

**Published:** 2022-02-11

**Authors:** Jun Li, Qingzhen He

**Affiliations:** ^1^Department of Emergency, Xi'an No. 3 Hospital, Xi'an 710018, China; ^2^Department of Endocrinology, Xi'an Gaoxin Hospital, Xi'an 710075, China

## Abstract

**Objective:**

Insulin replacement therapy is the main treatment method for type 1 diabetes, and adjuvant comprehensive treatment to reduce the complications of diabetes is still the focus of research. The purpose of this study is to explore the clinical efficacy of Tresiba combined with Ingredient Rehmannia Pill in the treatment of type 1 diabetes.

**Methods:**

A total of 216 patients with type 2 diabetes admitted to our hospital from January 2019 to July 2019 were enrolled in this study. Patients in the control and observation groups were treated with Tresiba and Tresiba combined with Ingredient Rehmannia Pill, respectively. The change of TCM symptom score, blood glucose level and fasting insulin level before and after treatment were evaluated, and the insulin resistance index was calculated to observe the adverse reactions of patients.

**Results:**

After treatment, the TCM syndrome scores of the two groups decreased significantly, and the TCM syndrome scores of the observation group were significantly lower than those of the control group. The fasting blood glucose, 2 h postprandial blood glucose and insulin resistance index of the observation group were lower than those of the control group. The levels of FBG, 2 hBG and HbA1C in the observation group were significantly lower than those in the control group. The total effective rate of the observation group was 91.7%, which was significantly higher than that of the control group (77.1%). The adverse reactions of patients in the observation group were slightly more than those in the control group.

**Conclusion:**

Our study demonstrated that Ingredient Rehmannia Pill combined with Tresiba is effective in the treatment of type 2 diabetes, providing alternative therapies for the treatment of diabetes.

## 1. Introduction

Diabetes is the most common metabolic disease, which is characterized by partial or complete destruction of pancreatic cells leading to insulin deficiency [1]. Diabetic patients have impaired pancreatic islet function at a young age and may require lifelong insulin therapy [2]. According to the report of the International Diabetes Federation, approximately 542,000 children worldwide suffer from diabetes [3]. In addition, about 86,000 children under the age of 15 suffer from diabetes each year, with an estimated annual incidence of 3% worldwide. Complications of diabetes, such as ketoacidosis, should cause widespread concern during the treatment process [4]. Ketoacidosis is still the most common complication after discharge from hospital in diabetic patients [5]. Although insulin replacement therapy is the main treatment method for diabetes, adjuvant comprehensive treatment to reduce the complications of diabetes is still the focus of future research.

The article "Evaluation of Tresiba Combined with Six Ingredient Rehmannia Pill in the Treatment of Type 2 Diabetes" was retracted in 2023. Reasons: signs of a paper mill; suspected computer-generated content; unreliable results or conclusions; lack of ethics approval or compliance.

Tresiba is a long-acting human insulin analogue suitable for blood glucose control in diabetic patients [6]. There is a risk of hypoglycemia when using insulin to treat diabetes. The ideal insulin should reduce the risk of hypoglycemia while controlling blood sugar [7]. At present, the long-acting insulin commonly used in clinical diabetes treatment mainly include insulin glargine and insulin dete. Tresiba is a new type of long-acting insulin analogue, which can act for more than 24 h [8]. Many clinical studies [9, 10] and observational studies [11, 12] have shown that degu insulin can effectively treat type 1 diabetes and improve the quality of life of patients [13]. However, these drugs are not effective in treating diabetic complications.

Six Ingredient Rehmannia Pill is a famous prescription of “nourishing Yin and strengthening kidney” in traditional Chinese medicine books. Previous studies have demonstrated that Six Ingredient Rehmannia Pill has the effects of lowering blood sugar, preventing diabetes and complications [14]. Six Ingredient Rehmannia Pill combined with valsartan capsule can significantly improve the treatment effect of diabetic nephropathy [15]. It also can assist xiaoke pill in the treatment of type 2 diabetes to improve the efficacy and reduce adverse effects [16]. However, the efficacy of Six Ingredient Rehmannia Pill in the treatment of type 2 diabetes needs to be further verified. This study aimed to clarify the clinical effects of Six Ingredient Rehmannia Pill in the treatment of type 2 diabetes and its complications.

## 2. Materials and Methods

### 2.1. General Information

A total of 216 patients with type 2 diabetes admitted to our hospital from January 2019 to July 2019 were enrolled and divided into control group and observation group. The control group included 108 patients: 52 males and 56 females. The average age was 29.2 ± 15.9 years old. The average course of disease was 7.52 ± 0.71 years. The average body mass index was 21.92 ± 2.63 kg/m^2^. The observation group consisted of 53 males and 55 females. Mean age was 24.2 ± 13.8 years old, the average course of disease was 8.42 ± 1.35 years. The average body mass index was 21.39 ± 2.71 kg/m^2^. There was no significant difference in gender, age, disease course and body mass index between the two groups (*P* > 0.05).

The article "Evaluation of Tresiba Combined with Six Ingredient Rehmannia Pill in the Treatment of Type 2 Diabetes" was retracted in 2023. Reasons: signs of a paper mill; suspected computer-generated content; unreliable results or conclusions; lack of ethics approval or compliance.

### 2.2. Inclusion and Exclusion Criteria

  Inclusion criteria: (1) the patient had symptoms of polydipsia, polyphagia, polyuria and other symptoms, such as easy to hunger, dry stool knot, red tongue, fear of heat, and upset, and fasting blood glucose was above 7.0 mmol/L. The patient was definitely diagnosed as diabetes; (2) good drug tolerance; (3) did not use glucocorticoids and other hormone drugs in the past month; (4) the patient is not insulin resistant; (5) the patients were informed and agreed to the study.
  Exclusion criteria: (1) patients who do not follow the doctor's advice to take drugs and test blood glucose and lipid; (2) patients with life-threatening serious complications during treatment; (3) patients with severe infectious diseases, renal failure, and immune system diseases; (4) combination of emotional tension and severe anxiety cannot cooperate; (5) women during lactation or pregnancy.

### 2.3. Treatment

Patients in the control group received routine Tresiba treatment with 0.4 U/kg once a day. Patients in the observation group were treated with Six Ingredient Rehmannia Pill (Henan Wanxi pharmaceutical co., LTD., specification: 240 pills, approval number: national drug approval Z41022128) orally three times per day and eight pills per time besides routine Tresiba treatment. Both groups were treated for 12 weeks.

### 2.4. Observation Indicators

According to the “Guiding Principles for Clinical Research of New Traditional Chinese Medicine” [17], the changes in TCM symptom scores before and after treatment were evaluated. Nine main syndromes: dry throat, dry mouth, heavy dizziness, sore waist and knees, chest tightness, chest pain, white and greasy tongue coating or less bitterness, heavy numbness of limbs, fatigue, fatigue, and obesity. These five symptoms include fever, insomnia and irritability, menstrual cramps or menstrual disorders, constipation, scaly skin and dryness. According to the severity of symptoms, the score was divided into four levels: none, mild, moderate, and severe. The main scores were 0, 2, 4, and 6 points, and the secondary scores were 0, 1, 2, and 3 points. The total score was 69 points. The blood glucose levels and fasting insulin levels before and after treatment were detected in the two groups, and the insulin resistance index was calculated. Insulin resistance index = (fasting insulin × fasting blood glucose)/22.5. The patient adverse reactions during treatment were observed. The fasting blood glucose, fasting blood glucose (FBG), 2 h postprandial blood glucose (2 HBG), and glycosylated hemoglobin (HbA1C) were detected before and after treatment.

The article "Evaluation of Tresiba Combined with Six Ingredient Rehmannia Pill in the Treatment of Type 2 Diabetes" was retracted in 2023. Reasons: signs of a paper mill; suspected computer-generated content; unreliable results or conclusions; lack of ethics approval or compliance.

All records are collected by our hospital and completed by trained and qualified investigators. Data management will be carried out under the guidance of medical statistics experts. To ensure the accuracy of the data, 2 data administrators will input and proofread the data.

### 2.5. Criteria for Therapeutic Effects

Significant effect was defined as the disappearance or improvement of clinical symptoms or signs, fasting blood glucose <7.2 mmol/L, and 2 h postprandial blood glucose <8.3 mmol/L. Effective was defined as significant improvement in clinical symptoms and signs, fasting blood glucose <10.0 mmol/L, and 2 h postprandial blood glucose <8.3 mmol/L. Ineffectiveness was defined as no improvement or aggravation of clinical symptoms and signs.

### 2.6. Data Analysis

SPSS 20.0 was used for statistical analysis. Quantitative data were used for independent *t*-test and qualitative data were used for *χ*^2^ test. *P* < 0.05 was considered statistically significant.

## 3. Results

### 3.1. Comparison of TCM Syndrome Scores between the Two Groups before and after Treatment

No significant differences in TCM syndrome scores between the two groups before treatment were observed (*P* > 0.05, Figure 1 and Table 1). However, the treatment decreased TCM syndrome scores of the two groups significantly, TCM score of the observation group was significantly lower than that of the control group (*P* < 0.05).

### 3.2. Comparison of Blood Glucose and Insulin Resistance Index before and after Treatment between the Two Groups (Mean ± Standard Deviation)

Before treatment, there were no significant differences in fasting blood glucose, 2 h postprandial blood glucose, and insulin resistance index between the control group and the observation group (*P* > 0.05). After treatment, the fasting blood glucose, 2 h postprandial blood glucose and insulin resistance index of the observation group were significantly lower than those of the control group (*P* > 0.05, Table 2).

### 3.3. Comparison of FBG, 2 hBG and HbA1C between the Two Groups before and after Treatment (Mean ± Standard Deviation)

As shown in Table 3, there was no significant difference in the levels of FBG, 2 hBG, and HbA1C before treatment between the two groups. After treatment, the levels of FBG, 2 hBG and HbA1C in the two groups decreased, and the levels of FBG, 2 hBG and HbA1C in the observation group were significantly lower than those in the control group (*P* < 0.05).

### 3.4. Comparison of Therapeutic Effect between the Two Groups

As shown in Table 4 and Figure 2, the total effective rate of patients in the observation group was 91.7%, which was significantly higher than that in the control group (77.1%) (*P* < 0.05).

The article "Evaluation of Tresiba Combined with Six Ingredient Rehmannia Pill in the Treatment of Type 2 Diabetes" was retracted in 2023. Reasons: signs of a paper mill; suspected computer-generated content; unreliable results or conclusions; lack of ethics approval or compliance.

### 3.5. Occurrence of Adverse Reactions During Treatment in the Two Groups

As shown in Figure 3, there were 3 cases of loose stools and 2 cases of anorexia the control group. The adverse reaction rate was 4.63% (5/108). In the observation group, there were 2 cases of nausea, 2 cases of headache, and 2 cases of bloating. The adverse reaction rate was 6.25% (6/108). The incidence of adverse reactions in the observation group was slightly higher than that in the control group (2 = 1.106, *P*=0.293).

## 4. Discussion

As a systemic metabolic disease, diabetes mellitus is mainly manifested as elevated blood sugar [18], which is mostly caused by insufficient insulin secretion or dysfunction [19]. Diabetes is an autoimmune disease mediated by T lymphocytes. The destruction of *β* islet cells leads to inflammation, which leads to an absolute lack of insulin secretion, requiring lifelong treatment with exogenous insulin [20]. At present, insulin replacement therapy is the main treatment method for diabetes, but adjuvant comprehensive treatment to reduce the complications of diabetes is also the focus of research.

Previous studies have found that the intervention of Six Ingredient Rehmannia Pill can delay or prevent the occurrence of type 2 diabetes [21], and can improve the inflammatory response and increase the inflammation by regulating the expression of related genes, regulating cell apoptosis, and inhibiting the symptoms of liver and kidney yin deficiency caused by diabetes [22, 23]. In addition, compared with the use of metformin alone, Six Ingredient Rehmannia Pill combined with metformin have fewer adverse reactions, and the therapeutic effect is significantly improved [24, 25]. In this study, although the scores of TCM syndromes in the control group and the observation group were significantly reduced after treatment, the scores of the observation group were significantly lower than those of the control group, indicating that the therapeutic effect of Six Ingredient Rehmannia Pill combined with insulin degu was better than that of Degu insulin alone. Six Ingredient Rehmannia Pill combined with acarbose has accurate curative effect in the treatment of type 2 diabetes mellitus [26] and can be widely used in clinical practice, which further supports the conclusions of this study.

In addition, the comparison of fasting blood glucose, 2 h postprandial blood glucose and hba1c levels between the two groups and the clinical efficacy showed that Six Ingredient Rehmannia Pill had a significant treatment effect on type 2 diabetes. Although Six Ingredient Rehmannia Pill combined with Tresiba have more adverse reactions than Tresiba alone, the difference was not significant.

The article "Evaluation of Tresiba Combined with Six Ingredient Rehmannia Pill in the Treatment of Type 2 Diabetes" was retracted in 2023. Reasons: signs of a paper mill; suspected computer-generated content; unreliable results or conclusions; lack of ethics approval or compliance.

Our research has some limitations. The sample size of this research was limited. In the future, it is necessary to conduct a larger sample size research to further verify the conclusions of this research. At the same time, this study was not to verify the efficacy of Six Ingredient Rehmannia Pill on all complications of diabetes, which needs to be further verified by future studies.

## 5. Conclusion

In summary, Six Ingredient Rehmannia Pill combined with Tresiba has a significant therapeutic effect on type 2 diabetes and has the potential for clinical application. This research provided a research foundation for the future research on the treatment of diabetes and its complications.

## Figures and Tables

**Figure 1:** Comparison of TCM syndrome scores before and after treatment between the two groups. ^*∗*^*P* < 0.05, compared with that before treatment; ^#^*P* < 0.05, compared with the control group.

**Figure 2:** Comparison of therapeutic effect between the two groups.

**Figure 3:** Occurrence of adverse reactions in the two groups.

**Table 1:** Comparison of TCM syndromes before and after treatment between the two groups (mean ± standard deviation).

Group	Number	Before	After	*T* value	*P* value
Observation	108	51.63 ± 6.73	12.65 ± 2.77	36.489	0.000
Control	108	51.87 ± 6.29	18.97 ± 3.46	32.219	0.000
*T* value		0.178	7.936		
*P* value		0.428	0.000		

**Table 2:** Comparison of blood glucose and insulin resistance index between the two groups before and after treatment.

Group	Fasting blood glucose (mmol/L)		2 h postprandial blood glucose (mmol/L)		Insulin resistance index	
	Before	After	Before	After	Before	After
Control	12.87 ± 1.24	6.35 ± 1.16	19.33 ± 3.27	7.87 ± 0.55	4.83 ± 0.84	2.83 ± 0.34
Observation	12.65 ± 1.37	5.12 ± 0.95	19.54 ± 3.35	6.35 ± 0.31	4.99 ± 0.78	2.27 ± 0.16
*T* value	1.165	5.667	0.163	17.002	0.911	10.691
*P* value	0.123	0.000	0.537	0.000	0.167	0.000

**Table 3:** Comparison of FBG, 2 hBG and HbA1C before and after treatment in the two groups.

Group	Number	Time	FBG (mmol/L)	2 hBG (mmol/L)	HbA_1_C (%)
Control	108	Before	8.53 ± 1.59	14.15 ± 3.52	9.73 ± 2.13
		After	7.25 ± 0.58	10.26 ± 1.33	8.18 ± 1.60
Observation	108	Before	8.95 ± 1.63	14.83 ± 3.69	10.37 ± 2.06
		After	6.84 ± 0.50	9.26 ± 0.54	6.58 ± 1.20
*t*_1_, *P*			5.31, <0.01	7.04, <0.01	4.08, <0.01
*t*_2_, *P*			10.16, <0.01	10.48, <0.01	11.09, <0.01
*t*_3_, *P*			1.35, >0.05	0.88, >0.05	1.56, >0.05
*t*_4_, *P*			6.70, <0.01	4.75, <0.01	5.53, <0.01

(1) comparison before and after treatment in the control group; (2) comparison before and after treatment in the observation group; (3) comparison between groups before treatment; (4) comparison between groups after treatment.

The article "Evaluation of Tresiba Combined with Six Ingredient Rehmannia Pill in the Treatment of Type 2 Diabetes" was retracted in 2023. Reasons: signs of a paper mill; suspected computer-generated content; unreliable results or conclusions; lack of ethics approval or compliance.

**Table 4:** Comparison of therapeutic effect between the two groups.

Group	Number	Excellent	Effective	Ineffective	Total effective rate
Control	108	40	34	22	77.1
Observation	108	56	32	8	91.7^*∗*^

^*∗*^ *P* < 0.05, compared with control group.

## Data Availability

The authors confirm that the data supporting the findings of this study are available within the article.
